# From sepsis to acute respiratory distress syndrome (ARDS): emerging preventive strategies based on molecular and genetic researches

**DOI:** 10.1042/BSR20200830

**Published:** 2020-05-04

**Authors:** Qinghe Hu, Cuiping Hao, Sujuan Tang

**Affiliations:** Department of Critical Medicine, Affiliated Hospital of Jining Medical University, Shandong 272011, P.R. China

**Keywords:** acute pulmonary edema, immune response, plasma genetic pre-diagnosis, proinflammatory signal interference, vascular permeability

## Abstract

A healthy body activates the immune response to target invading pathogens (i.e. viruses, bacteria, fungi, and parasites) and avoid further systemic infection. The activation of immunological mechanisms includes several components of the immune system, such as innate and acquired immunity. Once any component of the immune response to infections is aberrantly altered or dysregulated, resulting in a failure to clear infection, sepsis will develop through a pro-inflammatory immunological mechanism. Furthermore, the severe inflammatory responses induced by sepsis also increase vascular permeability, leading to acute pulmonary edema and resulting in acute respiratory distress syndrome (ARDS). Apparently, potential for improvement exists in the management of the transition from sepsis to ARDS; thus, this article presents an exhaustive review that highlights the previously unrecognized relationship between sepsis and ARDS and suggests a direction for future therapeutic developments, including plasma and genetic pre-diagnostic strategies and interference with proinflammatory signaling.

## Introduction

Due to the development of both overactivation of the innate immune response and immunosuppression, sepsis is considered a medical emergency characterized by severe immune dysregulation with a very complex immunopathogenesis. At the beginning of the host–pathogen interaction, the innate immune system is considered the first line of defense in the clearance of the infection [1]. However, if innate immune cells, such as endothelial cells (ECs) [2], and the cytokines/chemokines they release fail to clear the pathogen, the overactivation of innate immune system will induce the production of additional proinflammatory cytokines, including IL-1α, IL-6, TNF-α, IFN-γ, and granulocyte-monocyte colony stimulating factor (GM-CSF) [3–6]. During the pro-inflammatory stage of sepsis, the infiltration of various inflammatory cells, such as macrophages, neutrophils, dendritic cells (DCs), and T cells, is also responsible for the severe immune dysregulation induced by sepsis.

As a severe medical problem, sepsis has imposed a significant socioeconomic burden on patients and physicians in both pediatric and adult intensive care units. Sepsis is characterized as a life-threatening condition with a series of pathophysiological symptoms such as hypertension, leukocytosis/leukopenia, and hyper/hypothermia, according to the third international consensus definitions of sepsis [7]. All these symptoms are consequences of the dysregulated immune response to an infection, which induces systemic inflammation and systemic infection. Additionally, late in the progression of the systemic inflammatory response, the decreased resistance is responsible for the induction of disseminated intravascular coagulation, multi-organ dysfunction syndrome (MODS) and eventually leads to the death of the patients [8]. Some scholars postulate that septic shock is a subtype of sepsis characterized by cellular and metabolic abnormalities and particularly profound cardiopulmonary circulation dysfunction, which leads to a greater risk of death than sepsis alone. Severe sepsis is another stage of disease development that involves an elevated plasma lactate level or even lactic acidosis, oliguria, acute respiratory distress syndrome (ARDS) and mental disorder of the patients [9]. However, researchers have not yet elucidated the multifactorial mechanisms by which sepsis induces ARDS or why the inflammatory cytokine storm eventually induces diffuse alveolar damage and severe hypoxia.

In 1967, Ashbaugh et al*.* [10] initially came up with the term “adult respiratory distress syndrome’’ to describe hypoxia in patients. After they realized that this lung condition occurred in patients of all ages, they replaced “adult” with “acute,” resulting in the current term “ARDS.” Diffusing alveolar injury is considered the pathological hallmark, which is induced by endothelial cells dysfunction and local inflammation [11]. Since endothelial cells are the primary interface for the exchange of substances between the blood and tissues, the microvascular endothelial dysfunction of alveoli interferes with oxygen transport and exchange and subsequently leads to severe refractory hypoxia in most living patients with acute respiratory distress syndrome. Despite the presence other predisposing conditions that induce a systemic inflammatory response and the development of ARDS in patients, such as pneumonia, aspiration, trauma, pancreatitis or multiple transfusions, sepsis is the leading cause of ARDS and accounts for 32% of the etiology of ARDS [12]. Although sepsis and ARDS are heterogeneous according to their definitions, ARDS is considered a devastating complication of severe sepsis. Based on the clinical data, sepsis-associated ARDS has a lower incidence in patients (approximately 6–7% in Western countries) than sepsis or ARDS alone, but patients with sepsis-related ARDS exhibit worse clinical outcomes [13,14]. Through clinical observations, patients with sepsis-related ARDS displayed more significant dyspnea, as evidenced by the lower PaO_2_ /FiO_2_ ratios than in patients with non-sepsis ARDS. The extreme hypoxia is the main cause of high mortality rates in the intensive care unit (approximately 38.2%) [15]. Additionally, sepsis-associated ARDS also leads to a prolonged recovery of patients from lung injury, less successful withdrawal from mechanical ventilation and a slower rate of extubation [16,17]. Most treatment strategies for patients with the costly and deadly critical illnesses sepsis, ARDS and sepsis-induced ARDS are designed to relieve ventilation disorders via mechanical ventilation, in which positive end-expiratory pressure (PEEP) settings play an important role [18]. Nevertheless, the morbidity rate of ARDS associated with severe sepsis remains high, and the mortality rate of severe sepsis has reached 50% in some countries [19]. Currently, the management of ARDS is not specifically different form patients with sepsis, such as pharmacological approaches (neuromuscular blockers and steroids), and other treatments only regard the adequate delivery of oxygen to the tissue as a primary goal, which fails to recognize or predict the progression of ARDS in patients with sepsis, and unable to decrease the mortality rate of patients with sepsis [20–22]. Thus, a specific treatment for sepsis-induced ARDS is highly desired.

From this perspective, this review emphasizes the underlying relationship between the pathogenesis of sepsis and ARDS. First, we briefly discuss the underlying mechanisms of ARDS induced by sepsis at the cellular level, such as the increased permeability of pulmonary capillaries, the dysfunction of alveolar epithelial cells and the infiltration of neutrophils, macrophages, monocytes, and lymphocytes. Furthermore, we summarize the changes in gene expression in patients with sepsis-associated ARDS to provide a more solid foundation for developing therapeutic interventions and may predict the induction of ARDS and the treatment response. Finally, we highlight promising approaches to inhibit the development of uncontrolled inflammatory damage by targeting transcellular signaling pathways. The timely identification and treatment for the vicious cycle of sepsis-induced ARDS are urgently needed to decrease morbidity and mortality rates.

## At the cellular level, sepsis-induced inflammatory cells damage alveolar capillaries and epithelial cells, resulting in diffuse alveolar damage

Acute respiratory distress syndrome is not only a life-threatening critical condition but also an inflammatory disease, of which the critical event is known as some type of sudden damages to blood vessels mediated by an ‘irritating cause’, such as sepsis [23]. Consistent with the updated definition of sepsis by the NIH NHLBI Panel, who consider it a severe endothelial dysfunction syndrome induced by intravascular and extravascular infections that lead to reversible or irreversible injury to the microcirculation, ARDS is also one stage in the process of multiple organ failure characterized by the increased permeability of pulmonary epithelial and capillary endothelial cells, the influx of large numbers of alveolar macrophages and neutrophils and cell apoptosis [24]. The severe inflammatory responses induced by sepsis lead to acute pulmonary edema by altering vascular permeability, which constitutes the exudative phase of ARDS [25].

In response to the invading pathogens, immunological mechanisms are activated. Some scholars have described the inflammation induced by the immune response as disease-related network, in which several pathogen-derived components of innate immunity interact nonlinearly [26]. The activation of antigen-presenting cells (APCs) includes the up-regulation of monocytes, macrophages, dendritic cells and endothelial cells. These APCs are responsible for activating signaling pathways among immune cells to release inflammatory mediators (interleukin (IL)-1, IL-6, IL-8, tumor necrosis factor (TNF) α) and further amplify the inflammatory response [1,27]. Since the immune system of patients with sepsis has become dysregulated, the pro-inflammatory signaling accelerates vascular endothelial dysfunction and subsequently promotes the influx of more inflammatory cells, such as neutrophils, monocytes, macrophages, and lymphocytes and forms such a vicious pro-inflammatory circle. During this severe systemic inflammation, the hyperpermeability of the pulmonary microvasculature is primary injury caused by sepsis in the progression of ARDS, and thus alveoli are filled with a plasma exudate [28]. Moreover, along with the losses of alveolar epithelial cells, which are caused by sepsis-induced apoptosis and necrosis, the increased exudate in alveolar spaces leads to alveolar edema and the formation of a hyaline membrane [29] (Figure 1).

**Figure 1:** Schematic depicting the induction of sepsis-induced ARDS in the exudative phase Due to the severe inflammatory response induced by sepsis, a large number of inflammatory factors and immune cells infiltrate the alveoli and form a hyaline membrane.Then, during severe systemic inflammation, the swelling and necrosis of alveolar capillary endothelial cells lead to increased permeability of pulmonary capillaries and aggravate alveolar edema. Pulmonary edema is one of the characteristic signs of ARDS and is the most severe consequence of the exudative phase.

Diffuse alveolar damage is regarded as the histological hallmark of the first and acute phase of ARDS. Due to vascular leakage, alveolar epithelial damage and the accumulation of free fluid, the capacity for oxygen exchange decreases and leads to acute respiratory failure that subsequently develops into ARDS [30]. Thus, strategies targeting sepsis progression and cut the connection of the inflammatory network at an appropriate time to maintain the integrity of the vascular barrier integrity are urgently needed.

## At the genetic level, genetic testing makes facilitates the prediction of ARDS

According to the present understanding of the pathogenesis of ARDS, immunometabolism controls the development of inflammation in patients with sepsis-induced ARDS by regulating the function of immune cells [31]. Although, the discoveries and advances targeting immune cells as an alternative approach for ARDS therapy have been reported recently, improved outcome and decreased mortality rates in patients with sepsis-related ARDS have not been explicitly described [32,33]. Therefore, the altered expression of genes in the blood of neutrophils from patients with ARDS has received considerable attention. Current studies have estimated changes in the expression of more than 1500 genes over time during the immunological responses associated with the innate immune system [34–36].

Previous studies have primarily concentrated on using high-throughput gene profiling as a powerful tool for mining the transcriptomics date for critical pathways and genes, which provides insights for future pathogenesis research and the development of treatments for sepsis-associated ARDS [37,38]. In terms of gene expression, patients with ARDS and patients with sepsis show significant similarities. From the Gene Expression Omnibus (GEO) database, researchers chose patients with ARDS and patients with sepsis and separately analyzed the datasets of their blood polymorphonuclear neutrophils by using bioinformatics methods. As shown in a Venn diagram 220 differentially expressed genes (DEGs) overlapped between patients with ARDS and patients with sepsis [39]. More specifically, accumulating evidence reveals roles for that microRNAs (miRNAs) in various processes regulating inflammation regulation and immune responses, as these molecules inhibit the translation or degradation of mRNA to regulate the expressions of target genes [40]. The signaling cascade downstream of Toll-like receptors (TLRs) is a major pathway controlled by that miRNAs, such as miR-155, miR-125b, miR-223, let-7i, and let-7e [41]. Based on the investigation of miRNAs in sepsis [42]. Shilei et al. explored the association of miR-125a and miR-125b with the ARDS risk. The relative expression of miR-125a and miR-125b was increased in all patients with sepsis, but compared with patients with sepsis without ARDS, miR-125b was expressed at significantly higher level in patients with sepsis-induced ARDS, indicating the value of miR-125b in distinguishing patients with sepsis-induced ARDS from patients with sepsis [43].

Additionally, dysregulated inflammation is the leading cause of sepsis. During the development of sepsis, mitochondrial DNA, one of the damage-associated molecular patterns (DAMPs), is released into patients’ plasma [44,45]. Therefore, Faust et al. performed experiments to investigate the association of plasma mtDNA levels with sepsis-induced ARDS. The levels of mtDNA were not associated with non-sepsis ARDS, but the 48-h circulating mtDNA levels were significantly associated with the ARDS risk in patients with sepsis, which increased to approximately 60% in patients in the 95th percentile of plasma mtDNA levels [46]. These findings not only offer a reliable, supportive preclinical data for ARDS predictions but also suggest that Toll-like receptor 9 (TLR9), an inhibitor of a major mtDNA receptor [47,48], represents a potential target for the treatment of sepsis-associated ARDS.

Moreover, other potential non-genetic biomarkers for ARDS have been identified. For instance, significantly lower plasma citrulline levels, the nitric oxide synthase (NOS) substrate, have been observed in patients with sepsis-associated ARDS compared with the non-ARDS group [49]. In contrast, in patients with critical illness (including sepsis)-induced ARDS, levels of soluble programmed death receptor-1 (sPD-1) were elevated in both serum and bronchial alveolar lavage (BAL) fluid [50]. Based on these results, plasma citrulline and sPD-1 levels represent two diagnostic biomarkers for sepsis-associated ARDS, and they might serve as a regulatory target to monitor and prevent the development of ARDS.

## Transcellular signaling regulation: emerging therapeutic strategies for sepsis-related ARDS

According to the clinical statistics, the median time to the onset of critical illness-related ARDS is only 48 h after hospital admission [51]. Due to the small window of time for ARDS prevention, alternative approaches targeting potential pro-inflammatory regulatory pathways and a combination of antibiotics are urgently needed. By targeting nuclear signaling, a treatment that is commonly used in cancer therapy, the progression of inflammation and altered metabolism could be delayed, inhibited, or even averted. Thus, researchers provided insights into the regulation of transcellular signaling pathways for ARDS treatment and provided a strong experimental and theoretical basis for future target-based therapeutics. Pharmacological agonists/antagonists that modulate proinflammatory pathways have been explored in several studies (Table 1). Most studies examining the inhibition of the inflammatory response have been conducted using a rat model of cecal ligation puncture (CLP)-induced ARDS to evaluate the effects of different agonists/antagonists. For instance, BRL-44408 maleate decreased the expression of cytokines in alveolar macrophages and attenuated the phosphorylation of ERK1/2, p38MAPK, and p65, suggesting that the antagonism of α-AR down-regulates the ERK1/2, p38MAPK, and p65 pathways to subsequently alleviate inflammation-induced ARDS [52]. Additionally, the down-regulation of the TLR4/MyD88 signaling pathway positively correlates with the decreased levels of TNF-α, IL-1β, TLR4, TLR9, MyD88, and NF-κΒ [53]. After a pretreatment with the anti-TLR4 monoclonal antibody, TNF-α and IL-1β levels were reduced in the BAL fluid and peripheral blood, and the levels of TLR4, TLR9, MyD88, and NF-κΒ in macrophages were also decreased, resulting in a decrease in inflammatory infiltration and lung edema.

**Table 1:** The emerging transcellular signal regulation pathway and its pharmacological regulator in sepsis-associated ARDS

Pharmacological ↑ agonist/antagonist ↓	Target Regulator	Downstream mediator	Cytokine regulatory site or pathway
↓ BRL-44408 maleate	α-Adrenoceptor (α -AR)	Extracellular regulated protein kinase (ERK1/2); p38MAPK; p65	TNF‐α IL‐6 CXCL2/MIP‐2 [44]
↓ Anti-TLR4 monoclonal antibody	TLR4	TLR4/MyD88 signaling pathway) TNF-α, IL-1β, TLR4, TLR9, MyD88, and NF-κΒ	TNF-α, IL-1β, TLR4, TLR9, MyD88, NF-κΒ [45]
↑ Cytosporone B (CsnB)	Nuclear orphan receptor Nur77	Endothelin-1 (ET-1)	Phosphorylation of NF-B p65 and p38 MAPK [46]
↑ 6-Mercaptopurine (6-MP)		Endothelin-1 (ET-1)	c-Jun/AP-1 pathway [47]
↓ DIM-C-pPhOH, C-DIM8		/	C-DIM8 could deactivate Nur77 but hardly distributes in the lung, which makes the effect of C-DIM8 on ARDS rats remain unknown [46,52,53]

At the transcriptional level, several studies have postulated an interaction between the nuclear orphan receptor and endothelin-1 (ET-1). As a negative regulator, Nur77 is activated by cytosporone B (CsnB) and suppresses ET-1 expression by decreasing the lipopolysaccharide (LPS)-induced phosphorylation of NF-κΒ p65 and p38 MAPK, which relieved lung injury in a mouse model of ARDS [54]. Furthermore, in vascular endothelial cells, 6-mercaptopurine (6-MP) also activates Nur77and subsequently decreases ET-1 expression by inhibiting AP-1-dependent c-Jun promoter activity [55]. To date, several studies have highlighted factors that are associated with the underlying mechanism of ARDS onset (Table 2), of which the overexpression of miR-494 and lincRNA-p21 induces the pro-inflammatory response and lung fibroblast proliferation, respectively [56,57]. According to recent evidence, the up-regulation of sirtuin1 (SIRT1) mediated by the down-regulation of miR-199a suppresses excessive inflammatory responses and inhibits cellular apoptosis in rats with sepsis-induced ARDS [58]. All these future therapeutic targets exhibit the potential to negatively regulate ARDS progression in patients with sepsis; therefore, target-based therapeutic strategies and clinical trials are anticipated in the future.

**Table 2:** The potential regulatory targets and pathways for ARDS therapeutic strategies

Regulatory targets	Downstream mediator	Anti-ARDS pathway
MiR-494	NAD(P)H: quinone oxidoreductase 1 (NQO1);	In a rat model of sepsis-associated ARDS, the up-regulation of miR-494 decreased the expression of the antioxidant factor NQO1 and inactivated the Nrf2 signaling pathway, which were responsible for significantly higher levels of IL-1β, IL-6, and TNF-α, suggesting a pro-inflammatory effect of miR-494 on sepsis-associated ARDS [48].
miR-199a	Sirtuin1(SIRT1)	MicroRNA-199a (miR-199a) exerted a protective effect on sepsis-induced ARDS and was negatively correlated with SIRT1 expression. The down-regulation of miR-199a up-regulated SIRT1 expression, which suppressed excessive inflammatory responses and inhibited cellular apoptosis in subjects with sepsis-induced ARDS [50].
Jun N-terminal kinase (JNK) and p38	Mitogen-activated protein kinase (MAPK) signal	MAPK signaling is suppressed by blocking the phosphorylation of JNK and p38, which decreases the levels of the pro-inflammatory cytokines IL-6 and TNF-α and increases the level of the anti-inflammatory cytokine IL-10 to subsequently alleviate the inflammation in subjects with sepsis-induced ARDS [54].
RNFT2	IL-3Rα	RNFT2 decreases the expression of IL-3Rα by targeting it for proteasomal degradation after inducing its ubiquitination at Lys357, which inhibited pro-inflammatory cytokine and immune cell release in rats' lung inflammation models [55].
LincRNA-p21	Thy-1 (CD90)	The overexpression of lincRNA-p21 inhibits Thy-1 expression by inhibiting the acetylation of H3 and H4 at the Thy-1 promoter and remarkably suppressing the expression of the Thy-1 mRNA, which promotes the proliferation of the human lung fibroblasts cell line HLF1 [49].

## Conclusion

Currently, the overall treatment strategies for ARDS are not different from the treatments for patients with sepsis-induced ARDS, which mainly focuses on the adequate delivery of oxygen. Except for the prehospital use of aspirin or statins, drug-based preventive strategies do not exert a significant effect on reducing the development and mortality of severe sepsis-induced ARDS [59]. Thus, we certainly need a better understanding of the relationship between sepsis and ARDS to develop advanced treatments for sepsis-associated ARDS. Among the three major phases of ARDS pathogenesis, vascular hyperpermeability in the exudative phase remains a critical factor contributing to diffuse alveolar damage [60]. Moreover, the epithelial and endothelial cell damage induced by APCs-triggered immune responses also plays a crucial role in vascular leakage and alveolar edema. Therefore, many scholars hope to take the initiative to predict and prevent the occurrence and development of ARDS during the pro-inflammatory phase of sepsis. The release of many cytokine and the regulation of inflammatory pathways are regulated by some transcription factors such as NF-κB, thus, any changes in their structure and expression might influence cytokine production and ARDS progress [61]. Since increased IL-17 may serve as a biomarker to indicate the severity of ARDS in patients with sepsis-induced ARDS [62], researchers have estimated the IL-17 (rs763780, rs2275913, and rs8193036) and NF-κB1 (rs3774934) polymorphisms in a Chinese population that were associated with ARDS prediction and prognosis [63]. This conclusion further shows that the detection of related gene expression and variants has an important role in the prediction and prevention of the occurrence and development of ARDS. In critically ill patients, distant injury leading to subsequent lung failure is associated with DAMPs released by apoptotic cells [64], which are detected in plasma and enable clinicians to preliminarily diagnose ARDS in advance. In this review, we summarize the emerging plasma biomarkers for predicting and serving as targets to regulate sepsis-related ARDS. Although the molecular mechanisms regulating in the development of ARDS are complicated, many potential targetable mediators for sepsis-induced ARDS treatment exist. To date, several studies have explored the relationships between pharmacological agonists/antagonists and molecules regulating the onset of ARDS, but more studies are required to assess their efficiency and safety.

## Abbreviations

6-MP: 6-mercaptopurine
APC: antigen-presenting cell
ARDS: acute respiratory distress syndrome
BAL: bronchial alveolar lavage
CsnB: cytosporone B
DAMP: damage-associated molecular pattern
DC: dendritic cell
DEG: differentially expressed gene
EC: endothelial cell
ET-1: endothelin-1
GM-CSF: granulocyte-monocyte colony stimulating factor
IL: interleukin
LPS: lipopolysaccharide
miRNA: microRNA
NOS: nitric oxide synthase
PEEP: positive end-expiratory pressure
SIRT1: sirtuin1
sPD-1: soluble programmed death receptor-1
TLR: toll-like receptor
TNF: tumor necrosis factor
